The article "Sanzi Yangqin Decoction Alleviates Allergic Asthma by Modulating Th1/Th2 Balance: Coupling Network Pharmacology with Biochemical Pharmacology" was published in 2022. Journal: Evid Based Complement Alternat Med.

# Sanzi Yangqin Decoction Alleviates Allergic Asthma by Modulating Th1/Th2 Balance: Coupling Network Pharmacology with Biochemical Pharmacology

**DOI:** 10.1155/2022/9037154

**Published:** 2022-09-29

**Authors:** Wenpan Peng, Yong Xu, Yunhai Zhou, Juanjuan Wu, Guiqing Peng, Yanlan Gu, Xianmei Zhou, Mingzhi Pu

**Affiliations:** ^1^Suzhou TCM Hospital Affiliated to Nanjing University of Chinese Medicine, Suzhou 215000, China; ^2^School of Chinese Medicine, School of Integrated Chinese and Western Medicine, Nanjing University of Chinese Medicine, Nanjing, China; ^3^Department of Respiratory Medicine, Jiangsu Province Hospital of Chinese Medicine, Nanjing 210029, China

## Abstract

This study aimed to verify that Sanzi Yangqin Decoction (SYD) can relieve asthma in mice and explore the effect on TH1/Th2 balance. The targets of SYD and asthma were explored from the public database using various methods. The potential targets and signaling pathways were identified by KEGG enrichment analysis from DAVID database. Mice asthma models were established using OVA and aluminum hydroxide. Lung tissues of mice were stained with HE and Masson. The contents of IFN-*γ*, IL-4, and TNF-*α* in BALF and IgE in mouse serum were detected using ELISA. In addition, the changes in Th1 and Th2 cells of the spleen were detected by flow cytometry. Fourteen core targets including IL4, IFNG, and MMP9 were identified for the treatment of asthma by SYD. The content of IL-4 in the lung tissue and BALF was gradually decreased with the increase in SYD concentration, while the IFN-*γ* was gradually increased. The drug significantly reduced IgE levels in serum and TNF-*α* in BALF. The number of Th1 cells in the spleen increased, while Th2 cells decreased in a concentration-dependent manner. SYD can alleviate pulmonary inflammation, restore Th1/Th2 balance, and relieve asthma.

## 1. Introduction

Bronchial asthma (hereinafter referred to as asthma) is a chronic inflammatory disease of the airway involving a variety of cells and cellular elements. It is characterized by obvious heterogeneity [1], with airway inflammation and hyperresponsiveness as the main pathological features [2–4]. It is generally believed that chronic inflammation plays an important role in the occurrence and development of asthma [5, 6]. Asthma is also often accompanied by pulmonary eosinophilia and excessive IgE secretion [7, 8]. At present, the number of patients with asthma has exceeded 334 million globally [9]. In developed countries, the prevalence of asthma is stable or decreasing but rising rapidly in developing countries [2]. Studies have found that asthma is closely related to Th1/Th2 imbalance [10]. IFN-*γ* and IL-4, the representative cytokines secreted by Th1 and Th2 [11–13], can modulate Th1/Th2 balance in the body [14–17].

The article "Sanzi Yangqin Decoction Alleviates Allergic Asthma by Modulating Th1/Th2 Balance: Coupling Network Pharmacology with Biochemical Pharmacology" was published in 2022. Journal: Evid Based Complement Alternat Med.

Sanzi Yangqin Decoction (SYD) has often been applied to treat asthma clinically due to its efficacy in resisting inflammation, suppressing coughing, and relieving asthma [18, 19]. At present, there are few studies on the mechanism of SYD in the treatment of asthma. In this study, possible mechanisms of action of SYD were screened based on network pharmacology, followed by experimental evaluation (Figure 1). It points out the direction for the follow-up study on the molecular mechanism of SYD regulating Th1/Th2 balance, provides a good reference for the clinical application and pharmacological mechanism research of SYD in the treatment of asthma, and enriches the relevant research reports.

## 2. Materials and Methods

### 2.1. Databases

Twelve databases involved in the network pharmacological analysis are shown in Table 1.

### 2.2. Acquisition of Common Targets

Active ingredients and potential targets of SYD were retrieved from TCMSP, SEA, and SwissTargetPrediction. Disease-related targets were harvested from GeneCards, CTD, and TTD with “asthma” as the index term. Venn diagram of *R* language was used to map potential targets of SYD to disease-related targets to yield common ones.

### 2.3. Screening of Core Targets

Common targets were imported into STRING online analysis platform to plot a PPI diagram with the minimum confidence set to 0.9. The generated file “string interactions.tsv” was imported into Cytoscape for topological analysis. Common targets with a degree and betweenness centrality greater than mean values were screened as core targets.

### 2.4. Network Construction

The common targets, disease-related targets, and compounds contained in SYD were imported into Cytoscape to construct a drug-target-disease network to inform topological analysis.

### 2.5. Enrichment Analysis

To describe and annotate the functions of core targets and explore their biological processes and signaling pathways, we carried out an enrichment analysis on core targets screened out. This was based on the DAVID database, with the species limited to “*Homo sapiens*”. GO terms can be subdivided into three nonoverlapping ontologies: molecular function (MF), biological process (BP), and cellular component (CC). The KEGG enrichment analysis was conducted to screen out potential signaling pathways of SYD to treat asthma. The results of the enrichment analysis were determined under the screening condition of *P* < 0.05.

### 2.6. SYD Preparation

SYD, a Chinese medicine compound, composed of Fructus Perillae (10 g), Semen Sinapis Albae (10 g), and Semen Raphani (10 g). They are dry and mature seeds of *Raphanus sativus* L. and *Sinapis alba* L. and the fruit of *Perilla frutescens* (L.) Britt., a labiate plant. Ten times the amount of water was added and decocted twice. The extracted liquid was filtered and concentrated to 0.3 g/mL. The qualified liquid was stored at −20°C for reserve.

The article "Sanzi Yangqin Decoction Alleviates Allergic Asthma by Modulating Th1/Th2 Balance: Coupling Network Pharmacology with Biochemical Pharmacology" was published in 2022. Journal: Evid Based Complement Alternat Med.

### 2.7. Animals

Sixty 8-week-old female C57BL/6J mice (body weight: 20–25 g) were provided by Suzhou Xishan Biotechnology Co. Ltd. (license no.: SCXK (Shanghai) 2019–0004, certificate no.: 201903602, ethical code: 201903A007). They were adaptively raised in the SPF Laboratory Animal Room of the Animal Center, Nanjing University of Chinese Medicine for one week at the temperature of (22 ± (2)°C and humidity of (75 ± (5)% under a 12h:12 h light: dark cycle, with free access to clean water and food. The number of animals in each cage is 5.

### 2.8. Grouping and Modeling

Mice were randomized into the blank, model, and dexamethasone group, as well as low-dose, medium-dose, and high-dose SYD groups, with 10 mice per group. Mice in all groups except the blank group were treated with intraperitoneal injections of 0.2 mL mixed solution of OVA with aluminum hydroxide (10 *μ*g/0.1 mL) on days 1 and 14. Sensitized mice were placed in an atomizer on day 21 for atomization with normal saline containing 2.5% OVA, once a day for 30 min, for three successive weeks. Mice in the blank group were treated with intraperitoneal injections of normal saline and aerosol inhalation. One h before stimulation, mice were given dexamethasone (2 mg/kg) and SYD (15 g/kg, 30 g/kg, and 45 g/kg) by gavage. Mice in the blank and model groups were given normal saline by gavage (Figure 2). Blood was collected via an orbital bleed to prepare serum. At the end of the experiment, mice were sacrificed with cervical disconnection, the spleen was harvested to prepare the single-cell suspension, and the obtained lung tissue was stored at −80°C for future use. All operations complied with the regulations on the administration of laboratory animals.

### 2.9. Q-PCR Detection of Core Targets Screened Based on Network Pharmacology

Total RNA was extracted from the lung tissue using TRIzol reagent and reversely transcribed to cDNA. Total RNA with an OD260/OD280 between 1.8 and 2.0 was used for Q-PCR. Following the manufacturer's instructions, the pure RNA was reverse transcribed to cDNA using Prime-Script RT reagent kit with gDNA Eraser (Takara, Japan; 42°C 40 min, 85°C 5 min, 4°C store). The primers were designed by the software Primer Premier, as shown in Table 2. SYBR Green I nucleic acid gel stain was employed for Q-PCR. With GAPDH as the internal reference, 2^−ΔΔC*t*^ values were calculated as the relative expression levels of core target genes.

The article "Sanzi Yangqin Decoction Alleviates Allergic Asthma by Modulating Th1/Th2 Balance: Coupling Network Pharmacology with Biochemical Pharmacology" was published in 2022. Journal: Evid Based Complement Alternat Med.

### 2.10. Histopathological Examination

The fixed lung tissue was dehydrated with ethanol, routinely embedded in paraffin, and sliced into sections, which were stained with HE to observe the pathological changes under a microscope. The degree of inflammatory infiltration in the lung tissue was scored as follows: 0 point: no inflammatory cells; 1 point: focal infiltration of small amounts of inflammatory cells around the trachea or blood vessels and on the alveolar walls; 2 points: patchy or focal inflammatory cell infiltration around the trachea or blood vessels and on the alveolar walls, with the involving area less than 1/3 of the cross-sectional area of the lung; and 3 points: diffuse inflammatory cell infiltration around the trachea or blood vessels and in the lung interstitium, with the involving area reaching 1/3–2/3 of the cross-sectional area of the lung.

### 2.11. Detection of Related Indicators by ELISA

Bronchoalveolar lavage fluid (BALF) was collected by inserting a catheter into the right main bronchus and flushing 800 *μ*l of PBS in and out of the lungs three times (∼600 *μ*l recovered) [20]. The contents of IL-4, IFN-*γ*, and TNF-*α* in BALF and of IgE in serum were detected in strict accordance with the ELISA kit instructions.

### 2.12. Determination of IL-4 and IFN-*γ* in the Lung Tissue by Western Blot Assay

The total protein extracted from the lung tissue was quantified by the BCA method. From this, 25 *μ*g of protein was loaded into each gel sample hole, separated by 10% SDS-PAGE, and then transferred to the PVDF membrane, which was incubated with primary and secondary antibodies. After being visualized using ECL reagent in the dark for 30 s, the bands were exposed using the gel imaging system. The average grey value was calculated using Image J software, and the relative protein expression levels of IL-4 and IFN-*γ* were determined with *β*-actin as the internal reference.

### 2.13. Detection of Th1 and Th2 in the Spleen by Flow Cytometry

To determine the Th1/Th2 ratio in the spleen, we first prepared splenic single-cell suspension. With Brefeldin as the blocking agent, cells were incubated for 4 h with PMA and ionomycin to evaluate the Th1 and Th2 cells. After being permeabilized in Perm/Wash buffer solution in the dark for 20 min, the cells were incubated at 4°C in the dark with CD4-FITC, IFN-*γ*-PE, and IL4-PE antibodies for 30 min, and then detected by flow cytometry (BD, Accuri C6 Plus, events: 10000). Th2 cells were expressed by CD4^+^ and IL4^+^ and Th1 cells by CD4^+^ and IFN-*γ*^+^.

### 2.14. Statistical Analysis

The data were presented as mean ± standard error of mean (SEM). One-way ANOVA analysis with Kruskal–Wallis test was used for multiple comparisons where *n* ≤ 10 (when heteroscedasticity occurred, the Wilcoxon test was used). *P* < 0.05 indicated statistical significance levels are presented as ^*∗*^*P* < 0.05, ^*∗∗*^*P* < 0.01, and ^*∗∗∗*^*P* < 0.001(blank, *n* = 10; model, *n* = 7; SYD 15 g/kg, *n* = 8; SYD 30 g/kg, *n* = 8; SYD 45 g/kg, *n* = 9; dexamethasone, *n* = 9; The *N* value of each group in the western blot is 3). Data were analyzed using Graphpad Prism 8.

The article "Sanzi Yangqin Decoction Alleviates Allergic Asthma by Modulating Th1/Th2 Balance: Coupling Network Pharmacology with Biochemical Pharmacology" was published in 2022. Journal: Evid Based Complement Alternat Med.

## 3. Results

### 3.1. Active Ingredients of SYD

Twenty active ingredients were screened out under the conditions of bioavailability (OB) ≥ 30% and drug-likeness (DL) ≥ 0.18% (Table 3). OB is the fraction (%) of an administered drug that reaches the systemic circulation, and DL is the resemblance of a compound to the existing drugs.

### 3.2. Network Relationship

Database retrieval yielded 119 SYD targets and 1,030 asthma-related targets. The potential targets of SYD were mapped to the asthma-related targets. Sixty common targets were obtained, based on which, a Venn diagram was plotted (Figure 3(a)). The common targets were then imported into Cytoscape to construct the drug-target-disease network, which involved 72 nodes and 141 edges. The node size represents the value of the degree (Figure 3(b). Topological analysis revealed that the network centralization, heterogeneity, and density were 0.363, 1.605, and 0.041, respectively.

### 3.3. Enrichment Analysis

The 60 common targets were imported into STRING online analysis platform, and 14 core targets were screened out based on degree and betweenness centrality (Figure 4(a)). These were then subjected to enrichment analysis using the DAVID platform. GO enrichment analysis showed that SYD affected such BPs as cell proliferation and apoptosis, nucleic acid metabolism, and protein transcription and translation (Figure 4(b)). KEGG enrichment analysis revealed that SYD mainly acted on asthma-related signaling pathways (Figure 4(c)), with IL-4 and TNF-*α* being the main action targets in treating asthma (Figure 4(d)).

### 3.4. Alleviation of OVA-Induced Asthma by SYD

HE and Masson staining results showed that compared to the model group, SYD effectively alleviated inflammation and collagen deposition in the lung tissue of mice and was increasingly effective with an increase in drug concentration (Figure 5(a)). There was a significant difference between the inflammation score and positive area in Masson (Figures 5(b) and 5(c)). In addition, SYD significantly reduced the content of TNF-*α* in BALF of model group mice and alleviated the inflammatory response (Figure 5(d)).

The article "Sanzi Yangqin Decoction Alleviates Allergic Asthma by Modulating Th1/Th2 Balance: Coupling Network Pharmacology with Biochemical Pharmacology" was published in 2022. Journal: Evid Based Complement Alternat Med.

### 3.5. Effects of SYD on the Key Proteins Expression

Transcription and protein synthesis of core target genes, screened by network pharmacology, was detected by Q-PCR and the western blot assay. Results from Q-PCR showed that multiple genes in the core targets were differentially expressed, including IL4, IFNG, and MMP9 (Figure 6(a)). The results of western blot display that the content of IL-4 in the lung tissue was gradually decreased with the increase in SYD concentration, while the content of IFN-*γ* was gradually increased. Quantitative analysis of the proteins showed that the differences in relative protein expression levels were statistically significant (Figures 6(b) and 6(c)). The contents of IL-4 and IFN-*γ* in BALF were detected using ELISA kits. We found that the contents of IL-4 gradually decreased with an increase in drug concentration, while the contents of IFN-*γ* gradually increased (Figures 6(d) and 6(e)). Detection of IgE content in serum revealed that the IgE content gradually decreased with an increase in drug concentration (Figure 6(f)).

### 3.6. Th1/Th2 in the Spleen

The percent of CD4^+^ IL-4^+^ T cells (Th2) in the model group was higher than those in the normal group, while percentages of CD4^+^ IFN-*γ*^+^*T* cells (Th1) decreased significantly (Figures 7(b) and 7(d)). Flow cytometry showed that SYD increased the content of Th1 cells in the spleen but reduced the content of Th2 cells. Compared with the blank group, the Th1/Th2 ratio in the model group was significantly lower. Compared with the model group, the Th1/Th2 ratios in the medication groups were significantly higher (Figures 7(a) and 7(c)).

## 4. Discussion

In this study, 14 core targets of SYD for the treatment of asthma were identified based on network pharmacology. Enrichment analysis of core targets showed that SYD exerted therapeutic effects on asthma mainly by regulating IL-4-mediated differentiation of Th0 cells. The protective effect of SYD on OVA-induced asthma in mice was explored with dexamethasone as the control. In the initial stage of provocation, sneezing, and scratching were observed, while choking, shortness of breath, nodding breathing, and other asthma-specific manifestations were observed in the later stage of provocation, accompanied by reduced activity and dull hair. HE staining results showed that SYD effectively ameliorated the inflammatory cell infiltration around the bronchi and blood vessels of mice in the model group. Q-PCR showed that IL4, IFNG, and MMP9 genes were differentially expressed in the mouse lung tissue. Western blot assay indicated that SYD reduced the content of IL-4 and increased the content of IFN-*γ* in the mouse lung tissue. In addition, the detection of IFN-*γ* and IL-4 in BALF and IgE in mouse serum in each group showed that SYD significantly increased the content of IFN-*γ* and reduced the contents of IL-4 and IgE. IFN-*γ* and IL-4, as the representative cytokines secreted by Th1 and Th2, reflected the Th1/Th2 balance affected by SYD. In general, SYD can increase the Th1/Th2 ratio in asthmatic patients and restore it to normal balance.

The article "Sanzi Yangqin Decoction Alleviates Allergic Asthma by Modulating Th1/Th2 Balance: Coupling Network Pharmacology with Biochemical Pharmacology" was published in 2022. Journal: Evid Based Complement Alternat Med.

In the serum of asthmatic patients, Th1 cells are rare and Th2 cells are abundant [21–23]. The Th1/Th2 imbalance is mainly manifested as a Th2-dominant response [24]. The imbalance of CD4^+^T cell subsets (Th1/Th2) leads to the destruction of the tissue structure by immune cells which is an important pathogenesis of asthma [25, 26]. An important sign of Th1 and Th2 differentiation is the secretion of cytokines IL-4 and IFN-*γ* [27–29], as initial CD4^+^T cells (Th0) secrete almost no cytokines [30]. Th1 and Th2 cells are differentiated by the unstimulated Th0 cells [31]. Under the stimulation of IL-12, Th0 cells can be differentiated into Th1 and secrete cytokines IFN-*γ* and IL-2 [32–34]. IFN-*γ*, as a specific cytokine secreted by Th1, can activate macrophages, engulf the damaged tissue, and initiate bodily self-repair to fight against asthma [35, 36]. It can inhibit the differentiation of Th2 cells induced by IL-4 to maintain Th1/Th2 balance [37] and inhibit the generation of IgE. It promotes the synthesis of IgG and reduces the release of cellular inflammatory mediators to prevent asthma [38, 39]. Under stimulation by IL-4, Th0 can be differentiated into Th2 and secrete cytokines such as IL-4 and IL-13 [40, 41]. The representative IL-4 can bind to IL-4R on B cells to activate the JAK/STAT signal transduction system and promote B cells to produce specific IgE [42]. Through binding to mast cells, IgE can induce mast cell degranulation and histamine and leukotriene release [43]. The level of serum IgE, a core antibody mediating type I allergic reaction, is closely related to the severity of asthma [38]. Furthermore, IL-4 can also promote the expression of vascular cell adhesion molecules and allow eosinophilic granulocytes to accumulate and infiltrate the inflammatory site [41]. The commonly used drug dupilumab is a human-derived anti-IL-4Ra monoclonal antibody that can inhibit the binding of IL-4Ra to IL-4 and IL-13 and block the signaling pathways mediated by IL-4 and IL-13 [44].

After treating asthmatic mice with SYD, IFN-*γ* levels in the lung tissue and BALF were increased significantly with an increase in the drug concentration. The results in the high-dose group were similar to those in the dexamethasone group. Similarly, IL-4 decreased significantly in a dose-dependent manner. The abovementioned IFN-*γ* and IL-4 were taken as the marker cytokines secreted by Th1 and Th2. The results of flow cytometry suggested that SYD modulated the Th1/Th2 balance in the spleen to relieve asthma.

The article "Sanzi Yangqin Decoction Alleviates Allergic Asthma by Modulating Th1/Th2 Balance: Coupling Network Pharmacology with Biochemical Pharmacology" was published in 2022. Journal: Evid Based Complement Alternat Med.

With the development of molecular biology, research on the clinical prevention and treatment of asthma is gradually deepening. Current studies have shown that the imbalance of Th1/Th2 is closely related to the pathogenesis of asthma. The advantages of TCM in the regulation of Th1/Th2 balance are mainly reflected in the aspects of multilink, multitarget, and multiapproach. Through molecular biological methods, in-depth exploration of TCM is expected to bring a breakthrough for the clinical prevention of asthma. At present, the specific mechanism of TCM regulating the imbalance of Th1/Th2 response is not very clear, and the author's follow-up research will focus on it.

## 5. Conclusion

It was confirmed that SYD alleviated the inflammation of mice with asthma, increased Th1 cells and decreased Th2 cells in the spleen, and restored the Th1/Th2 balance to relieve asthma symptoms.

## Figures and Tables

**Figure 1:** The flow diagram of the study design.

**Figure 2:** The schematic time-course of inducing animal model of asthma, treatment, and splenocyte isolation.

**Figure 3:** Network relationship of SYD in the treatment of asthma. (a) The intersection of drug and disease targets, the yellow area represents the range of SYD, and the blue area represents the range of asthma. (b) The 60 common targets of SYD and asthma were imported into STRING to generate the network diagram. The node size represents the degree value. The larger the diameter, the more critical the node is in the network.

**Figure 4:** Core targets were screened and enrichment analysis was performed. (a) The screening process of core targets. (b) GO functional annotation of core potential targets of SYD. Biological processes (BP), cellular components (CC), and molecular functions (MF) were ranked according to −log (*P* values). (c) KEGG enrichment analysis for core targets of SYD. The color represented the −log (*P* values), and the size represented the gene count. (d) The signaling pathway of SYD in the treatment of asthma. The red node is the potential therapeutic target of the drug.

**Figure 5:** SYD reduced inflammatory cell infiltration in OVA-induced mice. (a) Hematoxylin-eosin and Masson staining showed inflammatory cell infiltration and collagen deposition of the lung tissues. (b and c) Inflammation scores and positive area in Masson were quantified. (d) ELISA was used to measure the total TNF-*α* content (pg/mL) in BALF of mice (blank, *n* = 10; model, *n* = 7; SYD 15 g/kg, *n* = 8; SYD 30 g/kg, *n* = 8; SYD 45 g/kg, *n* = 9; dexamethasone, *n* = 9).

The article "Sanzi Yangqin Decoction Alleviates Allergic Asthma by Modulating Th1/Th2 Balance: Coupling Network Pharmacology with Biochemical Pharmacology" was published in 2022. Journal: Evid Based Complement Alternat Med.

**Figure 6:** SYD reduced the expression of IL-4 and IFN-*γ* in the lung tissue of the mice with asthma. (a) The gene expression of the core targets was detected by Q-PCR. (b and c) Protein expression of IL-4 and IFN-*γ* in the lung tissues were detected by western blot. *β*-actin served as a reference gene. All experiments were repeated in triplicate to average. (d and e) ELISA was used to measure the total IL-4 and IFN-*γ* content (pg/mL) in BALF of mice. (f) ELISA was used to measure the total IgE content (ng/mL) in serum of mice (blank, *n* = 10; model, *n* = 7; SYD 15 g/kg, *n* = 8; SYD 30 g/kg, *n* = 8; SYD 45 g/kg, *n* = 9; dexamethasone, *n* = 9).

**Figure 7:** Flow cytometry of various CD4^+^ T cells subtypes including (a) in plot FSC and SSC, Th1 lymphocyte population between CD4 and IFN-*γ* markers were selected. Th1 in the group treated with SYD and dexamethasone in comparison with the untreated group increased. (b) Bar plot of the average percentage of CD4^+^ IFN-*γ*^+^ cells. (c) In plot FSC and SSC, Th2 lymphocyte population between the CD4 and IL-4 markers were selected. Th2 levels in the treated groups with SYD and dexamethasone compared with the untreated group decreased. (d) Bar plot of the average percentage of CD4^+^ IL-4^+^ cells (blank, *n* = 10; model, *n* = 7; SYD 15 g/kg, *n* = 8; SYD 30 g/kg, *n* = 8; SYD 45 g/kg, *n* = 9; dexamethasone, *n* = 9).

**Table 1:** Database used in the study.

Databases	Websites
Traditional Chinese medicine systems pharmacology database and analysis platform (TCMSP)	https://tcmspw.com/tcmsp.php
Similarity ensemble approach (SEA)	https://sea.bkslab.org
SwissTargetPrediction	https://www.swisstargetprediction.ch
STRING	https://string-db.org
PharmMapper	https://www.lilab-ecust.cn/pharmmapper/
Universal protein (UniProt)	https://www.uniprot.org/
The database for annotation, visualization and integrated discovery (DAVID)	https://David.ncifcrf.gov/
Comparative toxicogenomics database (CTD)	https://ctd.mdibl.org
Therapeutic target database (TTD)	https://bidd.nus.edu.sg/group/ttd/ttd.asp
GeneCards suite	https://www.genecards.org

**Table 2:** Q-PCR primer information.

Gene Symbols	Forward Primer	Reverse Primer
CASP3	ATGGAAGCGAATCAATGGACT	TGTACCAGACCGAGATGTCA
EGFR	CCCACTCATGCTCTACAACCC	TCGCACTTCTTACACTTGCGG
EGF	TGGATGTGCTTGATAAGCGG	ACCATGTCCTTTCCAGTGTGT
IL6	CCTGAACCTTCCAAAGATGGC	TTCACCAGGCAAGTCTCCTCA
TNF	CAGGCGGTGCCTATGTCTC	CGATCACCCCGAAGTTCAGTAG
TP53	AGCTGGTGTTGGTAGGCAGT	CCTCACCATCATCACACTGG
JUN	TTCCTCCAGTCCGAGAGCG	TGAGAAGGTCCGAGTTCTTGG
IL4	CCAACTGCTTCCCCCTCTG	TCTGTTACGGTCAACTCGGTG
MAPK1	GGTTGTTCCCAAATGCTGACT	CAACTTCAATCCTCTTGTGAGGG
VEGFA	GCACATAGAGAGAATGAGCTTCC	CTCCGCTCTGAACAAGGCT
MMP9	TGTACCGCTATGGTTACACTCG	GGCAGGGACAGTTGCTTCT
ALB	TGCAACTCTTCGTGAAACCTATG	ACATCAACCTCTGGTCTCACC
PPARA	AACATCGAGTGTCGAATATGTGG	CCGAATAGTTCGCCGAAAGAA
PTGS2	CTGGCGCTCAGCCATACAG	CGCACTTATACTGGTCAAATCCC
GAPDH	AGGTCGGTGTGAACGGATTTG	GGGGTCGTTGATGGCAACA

The article "Sanzi Yangqin Decoction Alleviates Allergic Asthma by Modulating Th1/Th2 Balance: Coupling Network Pharmacology with Biochemical Pharmacology" was published in 2022. Journal: Evid Based Complement Alternat Med.

**Table 3:** The information about SYD active ingredients.

PubChem CID	Molecule names	OB (%)	DL
**9548595**	Citrostadienol	43.28	0.79
**6506063**	Eicosatrienoic acid	41.64	0.20
**9602469**	(E)-(4-methylbenzylidene)-(4-phenyltriazol-1-yl)amine	57.87	0.19
**5280794**	Stigmasterol	43.83	0.76
**444899**	Arachidonic acid	45.57	0.20
**5280489**	Beta-carotene	37.18	0.58
**222284**	Beta-sitosterol	36.91	0.75
**5281331**	Spinasterol	42.98	0.76
**5282768**	Gondoic acid	30.70	0.20
**173183**	Campest-5-en-3beta-ol	37.58	0.71
**5366013**	2,6,10,14,18-Pentamethylicosa-2,6,10,14,18-pentaene	33.40	0.24
**5280445**	Luteolin	36.16	0.25
**5283640**	24-Methylidenelophenol	44.19	0.75
**5997**	CLR	37.87	0.68
**101690**	Cycloeucalenol	39.73	0.79
**65252**	Obtusifoliol	42.55	0.76
**5366854**	Icosa-8,11,14-trienoic acid methyl ester	44.81	0.23
**12303645**	Sitosterol	36.91	0.75
**5367326**	Icosa-11,14,17-trienoic acid methyl ester	44.81	0.23
**222284**	*β*-sitosterol	33.94	0.70

## Data Availability

The data used to support the findings of this study are available from the corresponding author upon request.
